The article "Improvement in Hemodynamic Responses to Metaboreflex Activation after One Year of Training in Spinal Cord Injured Humans" was published in 2014. Journal: Biomed Res Int.

# Improvement in Hemodynamic Responses to Metaboreflex Activation after One Year of Training in Spinal Cord Injured Humans

**DOI:** 10.1155/2014/893468

**Published:** 2014-04-07

**Authors:** Raffaele Milia, Silvana Roberto, Elisabetta Marongiu, Sergio Olla, Irene Sanna, Luca Angius, Pierpaolo Bassareo, Marco Pinna, Filippo Tocco, Alberto Concu, Antonio Crisafulli

**Affiliations:** ^1^Sports Physiology Laboratory, Department of Medical Sciences, University of Cagliari, Via Porcell 4, 09124 Cagliari, Italy; ^2^Unit of Cardiology and Angiology, Department of Medical Sciences, AOU University of Cagliari, 09042 Monserrato, Italy

## Abstract

Spinal cord injured (SCI) individuals show an altered hemodynamic response to metaboreflex activation due to a reduced capacity to vasoconstrict the venous and arterial vessels below the level of the lesion. Exercise training was found to enhance circulating catecholamines and to improve cardiac preload and venous tone in response to exercise in SCI subjects. Therefore, training would result in enhanced diastolic function and capacity to vasoconstrict circulation. The aim of this study was to test the hypothesis that one year of training improves hemodynamic response to metaboreflex activation in these subjects. Nine SCI individuals were enrolled and underwent a metaboreflex activation test at the beginning of the study (T0) and after one year of training (T1). Hemodynamics were assessed by impedance cardiography and echocardiography at both T0 and T1. Results show that there was an increment in cardiac output response due to metaboreflex activity at T1 as compared to T0 (545.4 ± 683.9 mL*·*min^−1^ versus 220.5 ± 745.4 mL*·*min^−1^, *P* < 0.05). Moreover, ventricular filling rate response was higher at T1 than at T0. Similarly, end-diastolic volume response was increased after training. We concluded that a period of training can successfully improve hemodynamic response to muscle metaboreflex activation in SCI subjects.

## 1. Introduction

During dynamic exercise, arterial blood pressure is regulated by the central nervous system through a balance between systemic vascular resistance (SVR) and cardiac output (CO) [1, 2]. In able-bodied (AB) subjects, effective integration exists between these cardiovascular parameters, and this results in the normal hemodynamic and blood pressure response observed during exercise. In spinal cord injured (SCI) individuals, there is a partial loss of nervous control over circulation, and this deficit may alter hemodynamics during effort [3–6]. It has been proposed that the absence of peripheral vasoconstriction below the level of the spinal lesion is in part responsible for the phenomenon, since this reduced capacity to vasoconstrict both the arterial and venous vessels impairs cardiac preload and afterload. As a consequence, reduced stroke volume (SV) and CO during exercise as compared to AB subjects are seen in SCI individuals [5–7].

Moreover, it has recently been found that control over the cardiovascular system in response to muscle “metaboreflex,” a cardiovascular reflex evoked by those afferent nerve endings in the muscle that are sensitive to accumulation of muscle metabolic end-products [8], is altered in these patients, as demonstrated by their reduced blood pressure increment to this reflex. This phenomenon is to be ascribed to an impaired capacity to elevate SVR and to enhance ventricular filling rate (VFR) and SV [3]. These findings strengthen the concept that, in SCI individuals, there is a dearrangement in cardiovascular control, and this fact may be partly responsible for their difficulty in achieving normal CO levels during exercise.

It has been reported that arm training is beneficial for SCI subjects, as it significantly improves maximal oxygen uptake (VO_2max_). Furthermore, it has been suggested that training may exert positive effects on the cardiovascular apparatus [7, 9]. In particular, it has been reported in SCI subjects that a short period of arm training can induce significant improvement in myocardial efficiency and SV, probably because some increase in cardiac preload takes place due to an increase in venous tone [10]. Moreover, it has been demonstrated that arm training resulted in increments in norepinephrine and epinephrine in response to exercise [11]. Therefore, we expected that training would result in enhanced capacity to vasoconstrict circulation and increase SVR and cardiac preload. Thus, we wondered whether one year of arm training would lead to significant improvements in hemodynamic responses to metaboreflex activation.

In view of these considerations, this study was devised to test the hypothesis that one year of arm training was effective in increasing blood pressure response to muscle metaboreflex in spinal cord injured humans by improving the capacity to constrict both arteriolar and venous beds, thereby enhancing vascular resistance, cardiac preload, and stroke volume.

## 2. Methods

### 2.1. Study Population

Nine SCI individuals (2 females and 7 males) with clinically complete spinal lesions between the fourth thoracic and the first lumbar tract were enrolled. The study was approved by the local ethical committee and conforms to the principles of the Declaration of Helsinki. Written informed consent was obtained from all participants before commencing the investigation. All patients underwent full medical examination during which the location and completeness of spinal cord transection were determined by neurological testing of the pattern of muscle paralysis, sensory defect, and deep tendon reflex. All were clinically stable (time since injury between 5 and 15 years) and no individual was involved in any exercise-training program. At the time of the study, 5 patients were on antibiotics for urinary tract infections and 7 were receiving oxybutynin for the treatment of neurogenic bladder. Mean ± standard deviation (SD) of age, height, and body mass was 41.2 ± 11.2 years, 169.1 ± 9.3 cm, and 68.6 ± 11.8 kg, respectively.

### 2.2. Experimental Design

At the beginning of the study (T0), patients underwent the following tests to assess physical capacity and metaboreflex activity.

#### 2.2.1. Incremental Exercise Test (IET)

Patients performed an incremental exercise test on an electromagnetically braked arm-crank ergometer (XT Pro Top 600, Technogym, Forlì, Italy) to assess maximum value in workload achievable (*W*_max⁡_). This test consisted of a linear increase in workload (10 W/min), starting from 20 W, at a cranking frequency of 60 rpm, up to exhaustion, taken as the point at which the subject was unable to maintain a cranking rate of at least 50 rpm. During the IET oxygen uptake (VO_2_), carbon dioxide output (VCO_2_), respiratory exchange ratio (RER), and pulmonary ventilation (Ve) were measured breath by breath by means of a metabolic measurement cart (MedGraphics Breeze, St. Paul, MN) calibrated immediately before each test.

#### 2.2.2. Metaboreflex Activation Test (MAT)

After IET (interval of at least three days), each subject underwent the following study protocol, randomly assigned to eliminate any order effect.

- Postexercise muscle ischemia session (PEMI session): it includes three minutes of resting, followed by three minutes of exercise, consisting of arm cranking at 30% of *W*_max⁡_, followed by three minutes of PEMI on the left arm induced by rapidly (in less than three seconds) inflating a tourniquet to 200 mmHg immediately following the exercise. The cuff was kept inflated for three minutes. Three minutes of recovery was further allowed after the cuff was deflated, for a total of six minutes of exercise recovery. This protocol was used in a previous investigation dealing with metaboreflex in both SCI individuals and normal subjects and it was shown to be able to trap the muscle metabolites in the exercising limb and to maintain stimulation of the metaboreceptors with a substantial increment in blood pressure [3, 12].
- Control exercise recovery session (CER session): the same rest-exercise protocol used for PEMI was performed followed by a controlled exercise recovery of six minutes without tourniquet inflation.

Sessions (a) and (b) were spaced by a 30-minute interval during which the subject rested in order to completely recover. Both IET and MAT tests were carried out in a temperature-controlled, air-conditioned room (22°C, relative humidity 50%).

Tests were repeated after one-year training (T1) consisting of 3–5 hours/week of arm cranking against a workload corresponding to 60% of *W*_max⁡_. The workload applied in the PEMI and CER sessions was adjusted taking into consideration the new level of *W*_max⁡_ reached by subjects after the period of training.

During MAT, hemodynamic variables were assessed by employing the method of impedance cardiography (NCCOM 3, BoMed Inc., Irvine, CA), which allows for continuous noninvasive cardiodynamic measuring. Previous research studies have used impedance cardiography in hemodynamic assessment during exercise in SCI subjects [3, 6, 13]. The Sramek-Bernstein equation [14] was employed to calculate beat-to-beat SV. Moreover, from impedance traces, preejection period (PEP) and ventricular ejection time (VET) were also calculated [15]. Diastolic time was measured by subtracting the sum of PEP and VET from the cardiac cycle total period and, by dividing SV by diastolic time, we obtained the ventricular filling rate (VFR), which is a measure of the mean rate of diastolic blood flux [16–18].

Heart rate was calculated as the reciprocal of the electrocardiogram R-R interval and CO was obtained by multiplying SV · HR. Subjects were also connected to a standard manual sphygmomanometer for systolic (SBP) and diastolic (DBP) blood pressure assessment, which was performed in the right arm by the same physician throughout all protocol sessions. To calculate mean blood pressure (MBP), the formula previously described by Moran and coworkers [19] which assesses MBP by taking into account changes in the diastolic and systolic periods was employed. Systemic vascular resistance (SVR) was obtained by multiplying the MBP/CO ratio by 80, where 80 is a conversion factor to change units to standard resistance units. End-diastolic volume (EDV) was also assessed by means of two-dimensional echocardiography (M5 Diagnostic Ultrasound System, Mindray Bio-Medical Electronics Co., Shenzhen, China) using a hand-held 3.5 MHz ultrasound probe. Measures were performed in the apical four-chamber position and EDV was determined from frame corresponding to the onset of the ECG QRS complex in at least three cardiac cycles. Volumes were calculated automatically by software using a conventional formula: 8*A* ^2^/3*πL*, where *A* was the left ventricular area and *L* was ventricular longest length [20]. The ventricular area was determined by tracing along the inner edge of the endocardial targets, and the length was obtained by measuring the distance from the left ventricular apex to the midpoint of the mitral annulus. Individual values in each beat were calculated as the average of three trials of the same beat; that is, each beat value was the average from 3 measures.

### 2.3. Data Analysis 

Mean ± SD of maximum values of workload (*W*_max⁡_), HR (HR_max⁡_), VO_2_ (VO_2max_), VCO_2_ (VCO_2max_), RER (RER_max⁡_), and Ve (Ve_max⁡_) reached by subjects during the IET tests were calculated as the average of the last 15 s of exercise. Values in hemodynamic parameters during PEMI and CER tests were averaged over one minute and the third minute of recovery (i.e., when a steady state was expected to be reached) was taken into account. To assess metaboreflex activity, the following procedure was employed: for each parameter, the difference between the PEMI and the CER test was calculated. This procedure allowed us to assess metaboreflex response, that is, the response due to metaboreflex activity [21]. The rationale behind this procedure lies on the fact that, during the CER test, hemodynamic parameters recovered towards baseline with a normal behaviour. Differently, during the PEMI test, hemodynamic parameters were affected by metaboreflex activation that induced an extra response which could be assessed by subtracting the CER from the PEMI quantity in the level of the measured variable. Differences in mean ± SD of hemodynamic variables at T0 and T1 were assessed by means of the two-way ANOVA for repeated measures (factors: condition and time) followed by Tukey post hoc test when appropriate. Differences in variables responses between tests conducted at T0 and T1 were assessed by *t*-test for paired data. Statistics were carried out utilising commercially available software (Graph-Pad, Prism). Statistical significance was set at a* P *value of <0.05 in all cases.

## 3. Results

All subjects completed the protocol and none complained of unbearable pain or discomfort during the periods of arm circulatory occlusion.  Table 1 shows that there was no difference in any of the hemodynamic parameters at rest between T0 and T1.  Table 2 demonstrates that, after the one-year period of training, patients reached higher levels in *W*_max⁡_ and VO_2max_ expressed both in absolute and indexed values.

Figures 1 to 3 show results of hemodynamic parameters along with their responses at the beginning and at the end of the study. Statistics revealed that HR was similar between conditions. However, HR response was significantly increased after one-year training. In detail, HR response (b) was −4.5 ± 10.2 bpm at T0 and +4.6 ± 5.9 bpm at T1. Stroke volume was increased at T1 as compared to T0. However, SV response (d) was unchanged after the period of training, as it was on average +1.7 ± 14.8 and +5.4 ± 8.9 mL at T0 and T1, respectively. (e) and (f) in Figure 1 show that absolute CO value was unaffected by the period of training. However, there was an increment in CO response at T1 as compared to T0. Indeed, this parameter reached a level of +545.4 ± 683.9 mL·min^−1^ at T1, whereas at TO it was −220.5 ± 745.4 mL·min^−1^ on average.

Figures 2(a) and 2(b) demonstrate that MBP was significantly lower at T1 with respect to T0. Moreover, its response was significantly increased after one-year training. At T0, the mean ± SD value in this parameter was −1.4 ± 4.3 mmHg, while at T1 was +9.5 ± 8.2 mmHg. (c) and (d) in Figure 2 illustrate that SVR decreased and that its response was unaffected by the period of training, since it was on average −47.9 ± 383.2 and −16 ± 246.6 dynes·s^−1^·cm^−5^ at T0 and T1, respectively. Statistics did not reveal any difference in absolute values of VFR between T0 and T1; however, its response was higher after training than at the beginning of the study (Figures 2(e) and 2(f)). This parameter achieved a level of +51.7 ± 50.1 mL·s^−1^ at T1, whereas it was −15.1 ± 35.3 mL·s^−1^ at T0.

Finally, Figure 3 shows that EDV was similar between conditions, but EDV response increased after training, reaching on average +7.2 ± 22.2 mL and +25.7 ± 19.3 mL at T0 and T1, respectively.

## 4. Discussion

The aim of this study was to test the hypothesis that hemodynamic response to muscle metaboreflex activation could be improved in spinal cord injured subjects with one-year training. We found that mean blood pressure response was significantly increased during metaboreflex after the period of training, and this fact was accompanied by enhancement of heart rate, cardiac output, ventricular filling rate, and end-diastolic volume responses. Moreover, an improvement in patients' absolute values of stroke volume and a reduction in the levels of blood pressure and systemic vascular resistance were observed. Furthermore, maximum oxygen uptake and workload achieved during arm-cranking exercise were significantly increased by the training programme. Taken together, these facts strengthen the concept that exercise exerts a beneficial effect on the cardiovascular apparatus of these individuals.

It is well known that control over the cardiovascular system, due to the loss of innervation below the level of the lesion, is altered in SCI individuals. These subjects have a reduced capacity to vasoconstrict both the arteriolar and venous beds. Hence, they cannot properly increase SVR and cardiac preload in response to effort. Furthermore, it has been reported they have altered responses to muscle metaboreflex activation as they are unable to increase SV, thereby explaining their reduced CO in this setting [3]. Yet, they also exhibited impaired capacity to increase SVR to compensate for the lack of CO enhancement. All these facts caused a blunted blood pressure during metaboreflex recruitment as compared to AB individuals [3].

Results from the present investigation suggest that exercise training is effective in ameliorating this hemodynamic scenario, as MBP response was significantly increased after one year of arm-cranking training. In our opinion, this was the result of two phenomena: enhanced HR and constant SV response, which together increased CO response and raised blood pressure despite the lack of SVR increase. It is to be noted that SV was kept constant notwithstanding the increment in HR, which would have reduced diastolic time and ventricular filling. This fact was to be ascribed to VFR response that was significantly improved after training, thereby increasing venous return and cardiac preload. Consistent with this view, EDV significantly increased after one year of training. It must not be forgotten that the capacity to increase venous return is crucial to achieve normal hemodynamic response during metaboreflex [22, 23]. Moreover, it has been reported that the inability to increase venous return during exercise is one of the key factors leading to abnormal cardiovascular response to exercise in SCI individuals. This cardiovascular abnormality has been reported several times and has been associated with a disturbed redistribution of blood during exercise due to the lack of sympathetic-mediated vasoconstriction below the level of the spinal cord lesion [5, 6, 13]. This fact impairs venous return and cardiac filling and in part explains the low SV during exercise shown by these patients.

It remains to be explained why the training program was effective in ameliorating hemodynamics. One possible explanation is that training induced some beneficial heart adaptation which in turn resulted in an ameliorated myocardial performance and cardiac preload. In accordance with this scenario, there are previous findings showing that training was capable of improving myocardial efficiency and SV in paraplegic individuals, probably because an enhancement in cardiac preload took place. This latter fact could be the consequence of an improved venomotor tone, which in turn increased venous return [10]. Moreover, it is well known that exercise training can enhance myocardial diastolic functions and that it may potentially reverse diastolic dysfunction associated with several pathologies such as myocardial hypertrophy and ischemia [24]. In particular, this latter mechanism is of particular interest and future studies conducted by using techniques such as tissue Doppler, which can investigate myocardial diastolic functions at tissue level, are needed to better clarify this point. In the present study, the diastolic heart volume assessment conducted by echocardiography did not allow assessing diastolic function at tissue level. Hence, our hypothesis that exercise training enhances diastolic function in SCI patients remains speculative.

Another possible explanation is that training could enhance the catecholamine response during effort. In fact, it has been found that training induced an increment in circulating norepinephrine and epinephrine during exercise in SCI individuals [11]. Therefore, it was likely that training resulted in an enhanced capacity to vasoconstrict circulation, thereby increasing the capacity to vasoconstrict the venous beds, reducing venous pooling, and increasing venous return and cardiac preload. Moreover, this mechanism could induce an elevation in HR response, as was actually observed in the present investigation.

However, it should be noted that no SVR increment was detected, and this fact appears in contrast to the supposed increment in circulating catecholamines. Another possible explanation was that exercise training ameliorated local mechanism involved in the control of vascular tone. One possible factor is the myogenic response to transmural pressure, which has been found to be more pronounced in SCI with respect to AB subjects [25]. This fact is believed to play a pivotal role in the orthostatic tolerance in these subjects and it compensates for the lack of sympathetic innervation below the level of the spinal lesion. It has been reported that the presence of non-*α*-adrenergic vasoconstriction represents a dominant contributor to blood pressure control in AB subjects [26]. Actually, it has been found during low body negative pressure that vasoconstriction still persists after *α*-adrenergic blockade. This fact indicates that, at least in the legs, it is possible to evoke a local vasoconstriction without any sympathetic activation. It has been suggested that this mechanism plays a pivotal role in mediating leg vasoconstriction in SCI subjects [25] and probably it represents the only suitable one for SCI individuals to challenge blood pressure changes. It is possible to speculate that one year of training improved the myogenic capacity to respond to transmural pressure. However, this hypothesis remains to be demonstrated since, to the best of our knowledge, there is no study available that focuses on the effect of physical training on myogenic response in paraplegic individuals.

It was then possible that a combination of central adaptation at the heart level (i.e., ameliorated diastolic functions) and of peripheral adaptations at vascular level (i.e., increased capacity to constrict the venous bed) was responsible for the beneficial effect of exercise training on the ameliorated hemodynamic response to the muscle metaboreflex of SCI subjects found in our study.

### 4.1. Limitations of the Study

One possible limitation of the present study is the lack of ventilatory parameters assessment during the metaboreflex test. However, in a previous study, ventilatory parameters were not significantly different between SCI subjects and controls and between PEMI and CER tests [3]. Another potential limitation is the lack of a control group, that is, a group of SCI subjects who did not undergo any training program. This was due to the fact that we found it difficult to enroll a sufficient sample size of control SCI individuals who did not perform any exercise-rehabilitation program before the study and who gave their consent to enter the study protocol employed in the present investigation. A final consideration is about the fact that the level of lesion of SCI subjects was not uniform, as it ranged from the fourth thoracic to the first lumbar tract. It is well known that, in SCI subjects, the critical level of lesion is T4, as sympathetic and vagal outflows to the heart and vagal afferents from the baroreceptors are preserved in lesions below this level. Therefore, cardiac autonomic control is intact, and HR can be modulated, whereas the vascular neural control is blunted in lower body vascular segments innervated by sympathetic preganglionic fibers leaving the medulla below T4 [4, 5]. In our study, we paid particular attention to avoiding recruiting subjects with lesions above T4. In fact, HR response was normal during the IET. Thus, even though the level of spinal cord injury was different among subjects, their capacity to increase HR was intact. The only difference among subjects was probably in the amount of circulation which could be constricted during the metaboreflex.

In conclusion, data from the present investigation provides evidence that, in spinal cord injured subjects, a period of training, along with increased physical capacity, can successfully improve hemodynamic response to muscle metaboreflex activation. In fact, after the training period, there had been a higher mean blood pressure and cardiac output response during metaboreflex with respect to baseline. This result was likely the consequence of an ameliorated ventricular filling rate and end-diastolic volume, which were probably due to an improved capacity to vasoconstrict the venous beds, thereby reducing venous pooling and increasing venous return. Moreover, increased diastolic and systolic functions of the trained heart cannot be ruled out. It remains to be seen whether this cardiovascular adaptation to training can be ascribed to an enhanced diastolic function of the heart, to an augmented level of circulating catecholamines, to enhanced myogenic response to transmural pressure at venous level, or to a combination of all these phenomena.

## Figures and Tables

**Figure 1:** Absolute values during the control exercise recovery (CER) and the postexercise muscle ischemia (PEMI) tests and response in heart rate (HR, (a) and (b)), stroke volume (SV, (c) and (d)), and cardiac output (CO, (e) and (f)) during the muscle metaboreflex at T0 and T1. Values are mean ± SD. The *P* values indicate the overall main effect of time. There was no interaction effect. *P < 0.05 versus T0.

**Figure 2:** Absolute values during the control exercise recovery (CER) and the postexercise muscle ischemia (PEMI) tests and response in mean blood pressure (MBP, (a) and (b)), systemic vascular resistance (SVR, (c) and (d)), and ventricular filling rate (VFR, (e) and (f)) during the muscle metaboreflex at T0 and T1. Values are mean ± SD. The *P* values indicate the overall main effect of time. There was no interaction effect. *P < 0.05 versus T0.

**Figure 3:** Absolute values during the control exercise recovery (CER) and the postexercise muscle ischemia (PEMI) tests and response in left end-diastolic volume (EDV, (a) and (b)) during the muscle metaboreflex at T0 and T1. Values are mean ± SD. *P < 0.05 versus T0.

**Table 1:** Absolute values of hemodynamic data at T0 and T1 during the rest periods preceding PEMI and CER tests.

		HR (bpm)	SV (mL)	CO (L·min^−1^)	MBP (mmHg)	SVR (dyne·sec·cm^−5^)	VFR (mL·s^−1^)	EDV (mL)
T0	Rest before PEMI	78.9 ± 15.3	56.2 ± 13.3	4.4 ± 1.5	86 ± 10.1	1693.8 ± 583.7	168 ± 75.2	125.5 ± 32.3
	Rest before CER	80.4 ± 12.9	54.5 ± 13.9	4.3 ± 1.3	87.5 ± 9.7	1736.5 ± 618.8	167.2 ± 68.3	131.2 ± 38.3

T1	Rest before PEMI	81.3 ± 10.3	57 ± 14.2	4.6 ± 1.4	84.9 ± 8	1592.5 ± 580.1	180.6 ± 73.4	128.6 ± 41.4
	Rest before CER	78.2 ± 14.1	63.1 ± 13	4.9 ± 1.4	84.9 ± 9.1	1495.7 ± 555.4	196.5 ± 86.5	122.4 ± 36.7

HR: heart rate, SV: stroke volume, CO: cardiac output, MBP: mean blood pressure, SVR: systemic vascular resistance, VFR: ventricular filling rate, and EDV: end-diastolic volume. Values are mean ± SD.

**Table 2:** Maximum values of work rate (*W*_max⁡_), heart rate (HR_max_), oxygen uptake (VO_2max_, expressed both in absolute and indexed values), carbon dioxide production (VCO_2max_), respiratory exchange ratio (RER_max_), and pulmonary ventilation (Ve_max_) reached during the cardiopulmonary test at the beginning of the study (T0) and after a period of one-year training (T1). Values are mean ± SD.

	T0	T1	*P* value
*W*_max⁡_ (W)	97.1 ± 8.8	110.6 ± 7.8	*P* < 0.05
HR_max_ (bpm)	169.4 ± 5.7	164.5 ± 9.5	*P* > 0.05
VO_2max_ (mL·kg^−1^·min^−1^)	20.1 ± 3.1	22.6 ± 2.7	*P* < 0.05
VO_2max_ (mL·min^−1^)	1381.7 ± 188.2	1565.4 ± 318.2	*P* < 0.05
VCO_2max_ (mL·min^−1^)	1806.7 ± 265.8	1829.7 ± 749.1	*P* > 0.05
RER_max_	1.31 ± 0.11	1.19 ± 0.45	*P* > 0.05
Ve_max_ (L·min^−1^)	63.9 ± 12.7	62.7 ± 12	*P* > 0.05
